The article "The association between obesity and vitamin D deficiency modifies the progression of kidney disease after ischemia/reperfusion injury" was published in 2022. Journal: Front Nutr.

# The association between obesity and vitamin D deficiency modifies the progression of kidney disease after ischemia/reperfusion injury

**DOI:** 10.3389/fnut.2022.952028

**Published:** 2022-11-17

**Authors:** Desiree Rita Denelle Bernardo, Daniele Canale, Mariana Moura Nascimento, Maria Heloisa Massola Shimizu, Antonio Carlos Seguro, Ana Carolina de Bragança, Rildo Aparecido Volpini

**Affiliations:** ^1^Laboratorio de Investigacao Medica 12, Faculdade de Medicina, Universidade de São Paulo, São Paulo, Brazil; ^2^Laboratorio de Investigacao Medica 12, Hospital das Clinicas HCFMUSP, Faculdade de Medicina, Universidade de São Paulo, São Paulo, Brazil

**Keywords:** chronic kidney disease, acute kidney injury, obesity, adipose tissue, vitamin D deficiency, inflammation, renal fibrosis

## Abstract

Acute kidney injury (AKI) alters renal hemodynamics, leading to tubular injury, activating pathways of inflammation, proliferation, and cell death. The initial damage caused to renal tissue after an ischemia/reperfusion (I/R) injury exerts an important role in the pathogenesis of the course of AKI, as well as in the predisposition to chronic kidney disease. Vitamin D deficiency has been considered a risk factor for kidney disease and it is associated with tubulointerstitial damage, contributing to the progression of kidney disease. Obesity is directly related to diabetes mellitus and hypertension, the main metabolic disorders responsible for the progression of kidney disease. Furthermore, the expansion of adipose tissue is described as an important factor for increased secretion of pro-inflammatory cytokines and their respective influence on the progression of kidney disease. We aimed to investigate the influence of vitamin D deficiency and obesity on the progression of renal disease in a murine model of renal I/R. Male Wistar rats underwent renal I/R surgery on day 45 and followed until day 90 of the protocol. We allocated the animals to four groups according to each diet received: standard (SD), vitamin D-depleted (VDD), high fat (HFD), or high fat vitamin D-depleted (HFDV). At the end of 90 days, we observed almost undetectable levels of vitamin D in the VDD and HFDV groups. In addition, HFD and HFDV groups presented alterations in the anthropometric and metabolic profile. The combination of vitamin D deficiency and obesity contributed to alterations of functional and hemodynamic parameters observed in the HFDV group. Moreover, this combination favored the exacerbation of the inflammatory process and the renal expression of extracellular matrix proteins and phenotypic alteration markers, resulting in an enlargement of the tubulointerstitial compartment. All these changes were associated with an increased renal expression of transforming growth factor β and reduced expression of the vitamin D receptor. Our results show that the synergistic effect of obesity and vitamin D deficiency exacerbated the hemodynamic and morphological changes present in the evolution of renal disease induced by I/R.

The article "The association between obesity and vitamin D deficiency modifies the progression of kidney disease after ischemia/reperfusion injury" was published in 2022. Journal: Front Nutr.

## Introduction

Over the last few decades, there has been a growing interest in risk factors related to the progression of kidney disease. This fact is due to the high prevalence of chronic kidney disease (CKD) and its high costs, as well as the risk of progression to end-stage renal disease (1–3). In addition to advanced age, gender, and family history, there are other traditional and common risk factors related to the progression of kidney disease, including diabetes mellitus (DM), hypertension, obesity, and cardiovascular diseases (CVD) (3–5). Furthermore, non-traditional risk factors such as hypovitaminosis D has been considered as an aggravating feature regarding the evolution of kidney disease (2, 6–9). It is well known that kidney diseases are accompanied by decreased levels of vitamin D (9, 10), which impair the crucial role of the kidney in vitamin D metabolism. As a consequence, hypovitaminosis D disarranges the regulation of numerous physiological activities, including the renoprotection performed by that hormone (9, 10).

An increasing number of studies have been demonstrating a relation between hypovitaminosis D and anthropometric status (11–15). In 2015, a meta-analysis showed that the prevalence of vitamin D deficiency in obese and overweight individuals was, respectively, 35 and 24% higher when compared to lean subjects (16). This association between body mass index (BMI) and hypovitaminosis D is also described in sunny countries. Unger et al. observed a high prevalence of hypovitaminosis D in healthy Brazilian adults and showed a negative association between serum levels of vitamin D and BMI (17). Corroborating those data, Bolland et al. suggested a possible link involving the sequestration and deposition of vitamin D in the adipose tissue and the lower sun exposure by choice and lifestyle (17, 18). Moreover, it has been described that hypovitaminosis D in obesity occurs independently of factors, such as age, ethnicity, gender, and sun exposure (16, 19). In the 1970s, Rosenstreich et al. experimentally showed that adipose tissue had a greater storage capacity for the different forms of vitamin D compared to other organs and tissues (20). In 2000, Wortsman et al. demonstrated a lower bioavailability of vitamin D in obese patients compared to eutrophic individuals after acute ingestion of ergocalciferol or phototherapy session (21).

The article "The association between obesity and vitamin D deficiency modifies the progression of kidney disease after ischemia/reperfusion injury" was published in 2022. Journal: Front Nutr.

It is acknowledged that adipose tissue is not just a fat reservoir, but a dynamic tissue involved in the production of adipokines, including leptin, adiponectin, tumor necrosis factor α (TNF-α), chemotactic protein for monocytes 1 (MCP-1), transforming growth factor β (TGF-β), angiotensin II (Ang II), and endothelin-1 (22, 23). This endocrine action of adipose tissue generates oxidative stress, activates the renin-angiotensin-aldosterone system (RAAS), and promotes insulin resistance with subsequent abnormal production/accumulation of lipids (23–25). In addition, obesity has been linked to inflammation and is considered a risk factor for a decline in renal function (25, 26). Based on the information regarding the low levels of vitamin D in the course of renal diseases and the impaired bioavailability of this hormone in obese individuals, we aimed to study the influence of vitamin D deficiency and obesity in rats submitted to renal ischemia-reperfusion injury (IRI).

## Materials and methods

### Animals

Male Wistar rats (*Rattus novergicus*), weighing 180–200 g, were provided by the animal facility from the Institute of Biomedical Sciences–University of São Paulo. During the 90-day protocol, we kept our animals at a controlled temperature (23 ± 1°C) with a light/dark cycle of 12/12 h. All the experiments followed our institutional guidelines and were approved by the local Research Ethics Committee (CEUA, registration 1438/2020).

### Diets

We used four different types of diet in this experimental protocol: (1) standard diet (20% protein, 70% carbohydrates, and 10% lipids); (2) standard diet depleted in vitamin D (20% protein, 70% carbohydrates, 10% lipids, and vitamin D-free); (3) high-fat diet (20% protein, 35% carbohydrates and 45% lipids); and (4) high-fat diet depleted in vitamin D (20% protein, 35% carbohydrates, 45% lipids, and vitamin D-free)—purchased from PragSoluções Biociências (Jaú, São Paulo, Brazil). The animals were placed in cages according to their diet, with free access to water.

### Experimental protocol

We allocated the rats to four groups according to each type of diet: Standard (SD, *n* = 8), fed the standard diet for 90 days; Vitamin D deficient (VDD, *n* = 9), fed the vitamin D-free diet for 90 days; High-fat (HFD, *n* = 10), fed the high-fat diet for 90 days; and High-fat vitamin D deficient (HFDV, *n* = 10), fed the high-fat vitamin D-free diet for 90 days. On day 45, all the rats were anesthetized with 2,2,2-tribromoethanol [250 mg/Kg body weight (BW)]. Subsequently, a suprapubic incision was made for induction of renal IRI by clamping both renal arteries for 45 min, followed by reperfusion.

The article "The association between obesity and vitamin D deficiency modifies the progression of kidney disease after ischemia/reperfusion injury" was published in 2022. Journal: Front Nutr.

### Analysis of urine samples

Before the clearance studies, all the rats were placed in individual metabolic cages, on a 12/12-h light/dark cycle, with free access to drinking water. We collected 24-h urine to assess urinary output and then centrifuged the samples to remove suspended material. We evaluated urinary protein excretion by colorimetric assay (Labtest Diagnóstica, Minas Gerais, Brazil).

### Anthropometry

On day 90, we evaluated anthropometric measurements in the animals under anesthesia just before the inulin clearance experiment. We used a sterile non-extensible measuring tape to assess: body length (cm), from the nostrils to the beginning of the tail (nose-to-anus); abdominal circumference (cm), taking the largest zone of the abdomen as the reference; and thoracic circumference (cm), immediately behind the foreleg (27, 28). We determined the BMI by dividing the body weight (g) by the body length squared (cm^2^) (29).

### Inulin clearance and hemodynamic studies

On day 90, we anesthetized the animals with sodium thiopental (50 mg/Kg BW) and then we cannulated the trachea with a PE-240 catheter for spontaneous breathing. The jugular vein was cannulated with a PE-60 catheter for infusion of inulin and fluids. To monitor mean arterial pressure (MAP) and collect blood samples, the right femoral artery was catheterized with a PE-50 catheter. We assessed MAP with a data acquisition system (MP100; Biopac Systems, Santa Barbara, CA). To collect urine samples, we cannulated the bladder with a PE-240 catheter by suprapubic incision. After the surgical procedure, a loading dose of inulin (100 mg/Kg BW diluted in 1 mL of 0.9% saline) was administered through the jugular vein. A constant infusion of inulin (10 mg/Kg BW) was started and continued at 0.04 mL/min throughout the whole experiment. We collected three urine samples at 30-min intervals. Blood samples were obtained at the beginning and at the end of the experiment. Inulin clearance values represent the mean of three periods. Plasma and urinary inulin were determined by the anthrone method, and the glomerular filtration rate (GFR) data were expressed as mL/min/100 g BW. To measure renal blood flow (RBF), we made a median incision and dissected the left renal pedicle for isolating the renal artery. An ultrasonic flow probe was placed around the exposed renal artery, and RBF was measured (mL/min) with an ultrasonic flow meter (T402; Transonic Systems, Bethesda, MD). We divided blood pressure by RBF to calculate renal vascular resistance (RVR, mmHg/mL/min).

### Biochemical parameters

We collected blood samples after the clearance studies to assess plasma levels of 25-hydroxyvitamin D [25(OH)D], parathormone (PTH), aldosterone, Ang II, total cholesterol (cholesterol), triglycerides, glucose, leptin, phosphate (P_*P*_), and calcium (P_*Ca*_). We assessed 25(OH)D, PTH, aldosterone, Ang II, and leptin by enzyme-linked immunosorbent assay (ELISA) using commercial kits: 25-hydroxyvitamin D (ALPCO, Salem, NH, USA); Rat Intact PTH (Immutopics, Inc., San Clemente, CA, USA); Aldosterone (Enzo Life Sciences, Farmingdale, NY, USA); Rat angiotensin II (Elabscience, Houston, TX, USA); Leptin (EMD Millipore, St. Louis, MO, USA). We measured P_*Ca*_, P_*P*_, and glucose by colorimetric assay (Labtest Diagnóstica, Minas Gerais, Brazil). Plasma levels of cholesterol and triglycerides were determined by specific electrodes (ABL800Flex—Radiometer, Brønshøj, Denmark).

The article "The association between obesity and vitamin D deficiency modifies the progression of kidney disease after ischemia/reperfusion injury" was published in 2022. Journal: Front Nutr.

### Tissue samples preparation

After the blood samples collection, we perfused the kidneys with a phosphate-buffered solution (PBS, pH 7.4). We froze the right kidneys in liquid nitrogen and stored them at –80°C for western blotting, ELISA, and real-time quantitative polymerase chain reaction (qPCR). The left kidneys were removed and a fragment of the renal tissue was fixed in methacarn solution (60% methanol, 30% chloroform, 10% glacial acetic acid) for 24 h and replaced by 70% alcohol thereafter. The kidney blocks were embedded in paraffin and cut into 4-μm sections for histological and immunohistochemical (IHC) studies.

### Total protein isolation

Kidney samples were homogenized in ice-cold isolation solution (200 mM mannitol, 80 mM HEPES, and 41 mM KOH, pH 7.5) containing a protease inhibitor cocktail (Sigma Chemical Company, St. Louis, MO, USA) with a homogenizer (Tissue Master TM125, Omni International, Kennesaw, GA, USA). Homogenates were centrifuged at 4,000 × rpm for 30 min at 4°C to remove nuclei and cell debris. Supernatants were isolated, and protein was quantified by Bradford assay (Bio-Rad Laboratories, Hercules, CA, USA).

### Western blot assay

For western blot analysis, 100 μg of total kidney protein was separated on SDS-polyacrylamide minigels by electrophoresis (30). After a transfer by electroelution to PVDF membranes (GE Healthcare Limited, Little Chalfont, UK), blots were blocked for 1 h with 5% non-fat milk in a Tris-buffered saline solution. Blots were then incubated overnight with a primary antibody for anti-VDR (1:500; Santa Cruz Biotechnology, Santa Cruz, CA, USA). The labeling was visualized with a horseradish peroxidase-conjugated secondary antibody (anti-mouse, 1:2,000; Sigma Chemical, St. Louis, MO, USA) and enhanced chemiluminescence detection (GE Healthcare Limited, Little Chalfont, UK). Kidney protein levels were further analyzed with a gel documentation system (Alliance 4.2; Uvitec, Cambridge, UK) and the software Image J for *Windows* (Image J-NIH Image). We used densitometry to quantitatively analyze the protein levels, normalizing the bands to β-actin expression (anti-β-actin, Sigma Chemical, St. Louis, MO, USA).

The article "The association between obesity and vitamin D deficiency modifies the progression of kidney disease after ischemia/reperfusion injury" was published in 2022. Journal: Front Nutr.

### Enzyme-linked immunosorbent assay in renal tissue

We assessed collagen type 3 (Col-3), Ang II, and MCP-1 in renal tissue by ELISA using commercial kits (Elabscience, Houston, TX, USA). The detection system and the quantification followed the protocols described by the manufacturer. The absorbances were obtained using the Epoch/2 device (Biotek Instruments, Winooski, VE, USA).

### Light microscopy

Four-μm histological sections of kidney tissue were stained with Masson’s trichrome and examined under light microscopy. We quantified the fractional interstitial area (FIA) by analyzing tubulointerstitial involvement and glomerular tuft area as well. For histomorphometry, the images obtained using microscopy were captured on a computer screen *via* an image analyzer software (ZEN, Carl Zeiss, Munich, Germany). For FIA evaluation, we analyzed 30–40 grid fields (0.09 mm^2^ each) per kidney cortex. The interstitial areas were manually demarcated, and the proportion of the field was determined after excluding the glomeruli. For the glomerular area, we calculated the arithmetic mean after analyzing approximately 80 glomeruli per kidney section. The glomerular tuft area (μm^2^) was manually circulated and automatically calculated by the software. We minimized bias during the morphometric analysis by keeping the observer blinded to the treatment groups.

### Immunohistochemical analysis

Immunohistochemistry was performed on 4-μm-thick paraffinized kidney sections mounted on 2% silane-coated glass slides. We used the following antibodies: mouse monoclonal to CD68 (ED1, 1:100; BioRad, Hercules, CA, USA); rabbit polyclonal to mannose receptor (CD206, 1:2,000; Abcam, Cambridge, MA, USA); mouse monoclonal to CD3 (1:50; Dako, Glostrup, Denmark); mouse monoclonal to α-smooth muscle actin (α-SMA, 1:200; Millipore, Billerica, MA, USA); rabbit monoclonal to fibronectin (1:400; Abcam, Cambridge, MA, USA); mouse monoclonal to vimentin (1:100; Dako, Glostrup, Denmark); rabbit polyclonal to TGF-β1 (1:100; Santa Cruz Biotechnology, Santa Cruz, CA, USA); mouse monoclonal to proliferating nuclear cell antigen (PCNA, 1:50; Dako, Glostrup, Denmark); and mouse monoclonal to JG12, direct against to aminopeptidase P (1:100; Santa Cruz Biotechnology, Santa Cruz, CA, USA). We subjected the kidney tissue sections to IHC reaction according to the protocol for each primary antibody. Reaction products were detected by anti-rabbit or mouse EnVision+ System™ and the color reaction was developed in 3,3-diaminobenzidine (Dako North America, Carpinteria, CA, USA). Counterstaining was with Harris’ hematoxylin. We analyzed 30–40 renal cortex fields (0.09 mm^2^) to evaluate the immunoreactions. The volume ratios of positive areas of renal tissue (%), determined by the color limit, were obtained by ZEN image analyzer software (Carl Zeiss, Munich, Germany) on a computer coupled to a microscope (Carl Zeiss Axioskop 40) and a digital camera (2, 31). To minimize bias during the IHC analysis, the observer was blinded to the treatment groups.

The article "The association between obesity and vitamin D deficiency modifies the progression of kidney disease after ischemia/reperfusion injury" was published in 2022. Journal: Front Nutr.

### Gene expression

We performed real-time qPCR in frozen adipose tissue assessing *VDR* gene (Rn00690616_m1). Firstly, we extracted and prepared total RNA by centrifugation technique using the commercial kit *SV Total RNA Isolation System* (Promega Corporation, Madison, WI, USA). Next, we determined the quantity and quality of RNA by Nanodrop™. We used 1 ul of RNA to prepare the cDNA following the manufacturer’s instructions of the *GoScript Reverse Transcription System* (Promega Corporation, Madison, WI, USA) and quantified again by Nanodrop™. We performed real-time PCR in 2 μl of cDNA (50 ng) using *GoTaq Probe qPCR Master Mix* (Promega Corporation, Madison, WI, USA) and *TaqMan on Step One Plus* (both from Applied Biosystems, Foster City, CA, USA). We evaluated relative gene expression with the 2^–ΔΔCt^ method (32) using glyceraldehyde 3-phosphate dehydrogenase (*GAPDH*) as the housekeeping gene (Rn01775763_g1).

### Statistical analysis

All data were expressed as mean ± SEM (standard error of the mean). Differences among groups were analyzed with GraphPad Prism 5.0 software (GraphPad Software, La Jolla, CA) by one-way analysis of variance followed by the Student–Newman–Keuls test. Values of *p* < 0.05 were considered statistically significant.

## Results

### Anthropometric parameters

We evaluated anthropometric data on day 90 of the experimental protocol. As expected, we observed a significant difference (*p* < 0.001) regarding the body weight of rats fed high-fat diets (HFD and HFDV) when compared to rats fed a standard diet (SD) or vitamin D-free diet (VDD) (Table 1). In addition, the body weight gain profile from HFD and HFDV groups reflected on the differences observed concerning the assessment of BMI (g/cm^2^), AC (cm), and TC (cm), as shown in Table 1. These results demonstrate that high-fat diets were effective in the experimental development of obesity. We did not find any difference in the length (cm) of the animals, characterizing a homogeneous and adequate growth in relation to the age and period studied (Table 1).

**TABLE 1:** Anthropometric parameters evaluated after the 90-day protocol in rats submitted to renal ischemia-reperfusion insult on day 45 treated with standard diet (SD), vitamin D-free diet (VDD), high-fat diet (HFD), or high-fat vitamin D-free diet (HFDV).

	SD	VDD	HFD	HFDV
Body weight (g)	425 ± 8	437 ± 10	531 ± 12^ad^	538 ± 16^ad^
BMI (g/cm^2^)	0.61 ± 0.01	0.61 ± 0.01	0.72 ± 0.02^ad^	0.72 ± 0.01^ad^
AC (cm)	17.4 ± 0.2	17.4 ± 0.3	21.5 ± 0.4^ad^	21.1 ± 0.4^ad^
TC (cm)	14.1 ± 0.3	13.9 ± 0.2	15.4 ± 0.2^ad^	15.4 ± 0.1^ad^
Length (cm)	26.4 ± 0.1	26.4 ± 0.1	26.8 ± 0.2	26.9 ± 0.1

BMI, body mass index; AC, abdominal circumference; TC, thoracic circumference.

The article "The association between obesity and vitamin D deficiency modifies the progression of kidney disease after ischemia/reperfusion injury" was published in 2022. Journal: Front Nutr.

Values are mean ± SEM. ^a^*p* < 0.001 *vs*. SD; ^d^*p* < 0.001 *vs*. VDD.

### Vitamin D, parathormone, and metabolic profile

We evaluated plasma concentration of 25(OH)D at 45 and 90 days of the protocol. We observed significantly lower levels (*p* < 0.001) of that hormone on day 45 in the animals that received vitamin D-depleted diets (VDD and HFDV) when compared to SD and HFD animals. These results confirm that those animals were deficient in vitamin D at the time they were submitted to renal IRI. As expected, we found almost undetectable levels of vitamin D in VDD and HFDV groups on day 90 (Figure 1). In addition, we noted that the HFD group presented sufficient but lower levels of vitamin D compared to the SD group (Figure 1). Although without significant differences among the groups, we observed an evident upward tendency in plasma levels of PTH (pg/mL) on day 90 in the vitamin D deficient groups (VDD and HFDV) in relation to SD and HFD groups (Table 2). We did not find any difference regarding plasma phosphate and calcium levels (data not shown).

**FIGURE 1:** Plasma 25(OH)D levels evaluated at 45 and 90 days of protocol in rats submitted to renal ischemia-reperfusion insult on day 45 treated with standard diet (SD), vitamin D-free diet (VDD), high-fat diet (HFD), or high-fat vitamin D-free diet (HFDV). Data are mean ± SEM. ^a^*p* < 0.001 *vs.* SD; ^d^*p* < 0.001 *vs.* VDD; ^g^*p* < 0.001 *vs*. HFD.

**TABLE 2:** Renal function, biochemical parameters, and glomerular tuft area evaluated after the 90-day protocol in rats submitted to renal ischemia-reperfusion insult on day 45 treated with standard diet (SD), vitamin D-free diet (VDD), high-fat diet (HFD), or high-fat vitamin D-free diet (HFDV).

	SD	VDD	HFD	HFDV
P_*PTH*_ (pg/mL)	464 ± 73	933 ± 187	552 ± 52	964 ± 176
C_*in*_ (mL/min/ 100 gBW)	0.64 ± 0.11	0.41 ± 0.05^c^	0.58 ± 0.02^f^	0.36 ± 0.02^bi^
UF (mL/24 h)	25 ± 2	16 ± 2^c^	18 ± 3^c^	15 ± 2^c^
Proteinuria (mg/24 h)	8.51 ± 0.50	9.65 ± 0.41	8.18 ± 0.71	10.83 ± 0.77^i^
RBF (mL/min)	6.06 ± 0.15	6.59 ± 0.15	5.20 ± 0.30^ce^	4.82 ± 0.22^bd^
RVR (mmHg/mL/ min)	21.26 ± 1.20	21.80 ± 0.95	23.67 ± 1.43	26.68 ± 0.88^cf^
GTA (μm^2^)	8934 ± 215	8927 ± 128	9230 ± 210	8670 ± 166

P_*PTH*_, plasma parathormone concentration; C_*in*_, inulin clearance; UF, urinary flow; RBF, renal blood flow; RVR, renal vascular resistance; GTA, glomerular tuft area. Data are mean ± SEM. ^b^*p* < 0.01 and ^c^*p* < 0.05 *vs*. SD; ^d^*p* < 0.001, ^e^*p* < 0.01 and ^f^*p* < 0.05 *vs*. VDD; ^i^*p* < 0.05 *vs*. HFD.

The article "The association between obesity and vitamin D deficiency modifies the progression of kidney disease after ischemia/reperfusion injury" was published in 2022. Journal: Front Nutr.

The analysis regarding lipid profile allowed us to observe isolated and synergistic actions of both high-fat and vitamin D-free diets on cholesterol and triglyceride levels. The evaluation of cholesterol levels (mg/dL) on day 90 showed a slight upward tendency in the VDD group in relation to the SD group. However, HFD group presented a significant increase concerning cholesterol levels compared to SD (*p* < 0.001) and VDD (*p* < 0.05) groups (Figure 2A). Furthermore, our results show that the vitamin D-free diet promoted a significant increase (*p* < 0.05) in triglyceride levels (mg/dL) in the VDD group compared to the SD group. We also observed higher and more significant triglyceride levels in the HFD group compared to the SD (*p* < 0.001) and VDD (*p* < 0.01) groups. Of note, the HFDV group presented higher levels of cholesterol and triglycerides in relation to all the other groups, demonstrating an evident imbalance of the lipid profile in vitamin D deficiency associated with obesity (Figure 2B). In addition, the results of fasting blood glucose (mg/dL) showed an upward tendency for this parameter in the VDD and HFD groups in relation to the SD group (Figure 2C). The animals from the HFDV group showed a noteworthy and significant increase in fasting blood glucose compared to all the other groups (Figure 2C). As expected, we observed a significant increase (*p* < 0.001) in plasma leptin levels (ng/mL) in the HFD and HFDV groups when compared to the SD and VDD groups (Figure 2D). This alteration was even more remarkable in the HFDV group, with a significant increase in comparison to all the other groups.

**FIGURE 2:** Plasma concentrations of **(A)** total cholesterol, **(B)** triglycerides, **(C)** glucose, and **(D)** leptin evaluated after the 90-day protocol in rats submitted to renal ischemia-reperfusion insult on day 45 treated with standard diet (SD), vitamin D-free diet (VDD), high-fat diet (HFD), or high-fat vitamin D-free diet (HFDV). Data are mean ± SEM. ^a^*p* < 0.001 and ^c^*p* < 0.05 *vs.* SD; ^d^*p* < 0.001, ^e^*p* < 0.01 and ^f^*p* < 0.05 *vs.* VDD; ^g^*p* < 0.001, ^h^*p* < 0.01 and ^i^*p* < 0.05 *vs*. HFD.

### Renal function and hemodynamic analysis

Our inulin clearance studies showed that the vitamin D-free diet associated or not with the high-fat diet modified the renal function. We observed a lower GFR (mL/min/100 g BW) in the VDD group (*p* < 0.05) compared to the SD group. This alteration was more evident in the HFDV group, which presented a lower GFR in comparison to the SD (*p* < 0.01) and HFD (*p* < 0.05) groups (Table 2). Regarding the urinary flow (mL/24 h), we found a lower urinary output (*p* < 0.05) in the VDD, HFD, and HFDV groups compared to the SD group (Table 2). In addition, we observed a slight upward tendency in proteinuria from VDD group in relation to SD and HFD groups and a significant increase (*p* < 0.05) of this parameter in the HFDV group compared to the HFD group (Table 2).

The article "The association between obesity and vitamin D deficiency modifies the progression of kidney disease after ischemia/reperfusion injury" was published in 2022. Journal: Front Nutr.

Our VDD, HFD and HFDV groups presented a higher MAP (mmHg) than the SD group. Supporting this data, we noticed a similar profile regarding plasma Ang II and aldosterone levels observed in the VDD, HFD, and HFDV groups in comparison to the SD group. Corroborating those findings, our results regarding the evaluation of renal expression of Ang II (pg/μg) showed an upward tendency in the amount of this polypeptide in the VDD, HFD, and HFDV groups in relation to the SD group. It is important to highlight that those alterations were more evident in the HFDV group (Figure 3).

**FIGURE 3:** **(A)** Mean arterial pressure (MAP), **(B)** plasma angiotensin II concentration, **(C)** quantitative amount of angiotensin II in renal tissue, and **(D)** plasma aldosterone concentration evaluated after the 90-day protocol in rats submitted to renal ischemia-reperfusion insult on day 45 treated with standard diet (SD), vitamin D-free diet (VDD), high-fat diet (HFD), or high-fat vitamin D-free diet (HFDV). Data are mean ± SEM. ^a^*p* < 0.001 and ^c^*p* < 0.05 *vs*. SD; ^f^*p* < 0.05 *vs*. VDD; ^i^*p* < 0.05 *vs*. HFD.

We also observed the influence of high-fat diets regarding RBF and RVR. HFD and HFDV groups presented a lower RBF (mL/min) than SD and VDD groups (Table 2). In addition, the HFD group showed a slight upward tendency in the RVR (mmHg/mL/min), while the HFDV group presented a significant increase (*p* < 0.05) of this parameter in relation to SD and VDD groups (Table 2).

### Vitamin D receptor expression and inflammation

We evaluated VDR protein expression in kidney tissue and VDR gene expression in the adipose tissue at the end of the 90-day protocol. The renal protein expression of VDR (%) was lower (*p* < 0.001) in the groups of animals that received the vitamin D-free diets (VDD and HFDV) when compared to the SD group (Figures 4A,B). Even with vitamin D deficiency, we observed a higher renal expression (*p* < 0.01) of VDR in the HFDV group than in the VDD group (Figures 4A,B). In addition, our results regarding real-time qPCR showed a downward tendency in VDR gene expression (ΔΔCt) in the adipose tissue from HFD and HFDV groups in relation to the SD group. Also, we noticed a significantly lower (*p* < 0.001) gene expression of VDR in the VDD group when compared to the SD group (Figure 4C).

The article "The association between obesity and vitamin D deficiency modifies the progression of kidney disease after ischemia/reperfusion injury" was published in 2022. Journal: Front Nutr.

**FIGURE 4:** Semiquantitative immunoblotting for renal vitamin D receptor (VDR) protein expression and RT qPCR for adipose tissue VDR gene expression evaluated after the 90-day protocol in rats submitted to renal ischemia-reperfusion insult on day 45 treated with standard diet (SD), vitamin D-free diet (VDD), high-fat diet (HFD), or high-fat vitamin D-free diet (HFDV). **(A)** Densitometric analysis of samples from an SD, VDD, HFD, and HFDV rat. **(B)** Representative immunoblots reacted with anti-VDR revealing a 51 kDa band. **(C)** Bar graph of VDR gene expression values. Data are mean ± SEM. ^a^*p* < 0.001 *vs*. SD; ^d^*p* < 0.001, ^e^*p* < 0.01 and ^f^*p* < 0.05 *vs.* VDD; ^h^*p* < 0.01 *vs*. HFD.

It is well known that vitamin D and adipose tissue are closely related to inflammation status. Based on that, we firstly evaluated the renal amount of MCP-1 (ng/μg protein) by ELISA and the renal expression of CD3+ and CD68+ cells (T cells and macrophages, respectively) by IHC studies (%). As shown in Figure 5A, we found a higher MCP-1 amount (*p* < 0.001) in the renal tissue from VDD and HFD compared to the SD group. This alteration was more evident in the HFDV group, which showed a significant increase in the renal amount of MCP-1 when compared to all the other groups (Figure 5A). Similarly, Figures 5B,C show a higher renal expression of CD3+ cells (*p* < 0.001) in the HFDV compared to all the other groups. Our next step was focused on the macrophage infiltration in the renal cortex. By using an anti-CD68 antibody we immunolocalized the M1 and M2 macrophages, also known to express the glycoprotein ED1 on their lysosomal membrane (33). As illustrated in Figures 6A,D, we observed a higher expression of CD68+ cells (*p* < 0.05) in the renal cortex from the VDD, HFD, and HFDV groups when compared to the SD group. Furthermore, for knowledge and differentiation between the macrophage subtypes, we evaluated the proportion of CD206+ cells (M2 macrophages) in relation to the whole amount of macrophages stained with CD68 (M1+M2 macrophages, Figure 6C). CD206 is also known as mannose receptor, which is an exclusive marker for M2 macrophages (1, 34). Although without significance among the groups, we observed a downward tendency in the expression of CD206+ cells in the VDD, HFD, and HFDV groups in relation to the SD group (Figures 6B,E), reinforcing the role of vitamin D and adipose tissue on the modulation of renal inflammation.

The article "The association between obesity and vitamin D deficiency modifies the progression of kidney disease after ischemia/reperfusion injury" was published in 2022. Journal: Front Nutr.

**FIGURE 5:** Quantitative amount of monocyte chemotactic protein 1 (MCP-1)—ELISA and immunohistochemical analysis for CD3+ cells (T cells) expression in renal tissue evaluated after the 90-day protocol in rats submitted to renal ischemia-reperfusion insult on day 45 treated with standard diet (SD), vitamin D-free diet (VDD), high-fat diet (HFD), or high-fat vitamin D-free diet (HFDV). **(A)** Bar graphs of MCP-1 quantification and **(B)** CD3+ cells expression values. **(C)** Representative photomicrographs of immunostaining for CD3+ cells in the renal cortex from an SD, VDD, HFD, and HFDV rat (×400). Data are mean ± SEM. ^a^*p* < 0.001 *vs.* SD; ^d^*p* < 0.001 *vs.* VDD; ^g^*p* < 0.001 and ^h^*p* < 0.01 *vs*. HFD.

**FIGURE 6:** Immunohistochemical analysis for CD68+ cells (M1 + M2 macrophages) and CD206+ cells (M2 macrophages) expression in the renal cortex evaluated after the 90-day protocol in rats submitted to renal ischemia-reperfusion insult on day 45 treated with standard diet (SD), vitamin D-free diet (VDD), high-fat diet (HFD), or high-fat vitamin D-free diet (HFDV). **(A)** Bar graph of CD68+ cells expression values. **(B)** Bar graph of CD206+ cells expression values. **(C)** Bar graph regarding the proportion of CD206+ cells in relation to the amount of CD68+ cells. Representative photomicrographs of immunostaining for CD68+ **(D)** and CD206+ **(E)** cells in the renal cortex from an SD, VDD, HFD, and HFDV rat (×400). Data are mean ± SEM. ^c^*p* < 0.05 *vs.* SD.

### Synergistic effect of vitamin D deficiency and adipose tissue on the renal expression of transforming growth factor β1 and extracellular matrix proteins

High-fat diets and hypovitaminosis D seem to be associated with the susceptibility to renal fibrosis formation (RFF) through an increased expression of TGF-β and extracellular matrix (ECM) components (1, 2, 35–37). In this study, we could observe the isolated influence of vitamin D deficiency and obesity, which contributed to a higher renal expression of TGF-β1 (%) in the VDD and HFD groups than in the SD group (*p* < 0.01). Simultaneously, we noticed a synergistic influence of both risk factors, which promoted a significant increase (*p* < 0.001) in the expression of TGF-β1 in the HFDV group compared to all the other groups (Figure 7).

**FIGURE 7:** Immunohistochemical analysis for transforming growth factor β1 (TGF-β1) expression in the renal cortex evaluated after the 90-day protocol in rats submitted to renal ischemia-reperfusion insult on day 45 treated with standard diet (SD), vitamin D-free diet (VDD), high-fat diet (HFD) or high-fat vitamin D-free diet (HFDV). **(A)** Bar graph of TGF-β1 expression values. **(B)** Representative photomicrographs of immunostaining for TGF-β1 in the renal cortex from an SD, VDD, HFD, and HFDV rat (×400). Data are mean ± SEM. ^a^*p* < 0.001 and ^b^*p* < 0.01 *vs*. SD; ^d^*p* < 0.001 *vs.* VDD; ^g^*p* < 0.001 *vs.* HFD.

The article "The association between obesity and vitamin D deficiency modifies the progression of kidney disease after ischemia/reperfusion injury" was published in 2022. Journal: Front Nutr.

To assess the production and secretion of ECM components generated from fibroblast activation, we investigated the renal expression of two ECM proteins, including Col-3 and fibronectin. First, our results showed a slight upward tendency in the renal amount of Col-3 (ng/μg) and a higher expression of fibronectin (%) in the VDD group in relation to the SD group. Meanwhile, the HFD group presented a higher renal expression of Col-3 and fibronectin than the SD group. Of note, those alterations were even more pronounced in the HFDV group. This group not only presented a higher amount of Col-3 in relation to SD and VDD groups, but also a significant increase in fibronectin expression compared to SD and HFD groups (Figure 8).

**FIGURE 8:** Quantitative amount of collagen 3—ELISA and immunohistochemical analysis for fibronectin expression in the kidney tissue evaluated after the 90-day protocol in rats submitted to renal ischemia-reperfusion insult on day 45 treated with standard diet (SD), vitamin D-free diet (VDD), high-fat diet (HFD), or high-fat vitamin D-free diet (HFDV). Bar graphs of **(A)** collagen 3 and **(B)** fibronectin expression values. **(C)** Representative photomicrographs of immunostaining for fibronectin in the renal cortex from an SD, VDD, HFD, and HFDV rat (400×). Data are mean ± SEM. ^a^*p* < 0.001, ^b^*p* < 0.01 and ^c^*p* < 0.05 *vs.* SD; ^e^*p* < 0.01 *vs*. VDD; ^i^*p* < 0.05 *vs*. HFD.

### Obesity and vitamin D deficiency increase the phenotypic change of renal cells

We studied the presence of markers of phenotypic change which included the renal expression of α-smooth muscle actin (α-SMA) and vimentin. We observed a mild upward tendency in the renal expression of α-SMA and a significant increase (*p* < 0.05) in vimentin expression in the VDD group in relation to the SD group. Simultaneously, we noticed a higher α-SMA expression (*p* < 0.05) and a slight upward tendency in vimentin expression in the HFD group compared to the SD group. Regarding the HFDV group, we found a higher vimentin expression than the SD group and a significant increase in renal expression of α-SMA compared to all the other groups (Figures 9, 10). Based on our results, it is plausible to suggest that the synergistic effect of vitamin D deficiency and obesity increased the phenotypical change of renal cells.

The article "The association between obesity and vitamin D deficiency modifies the progression of kidney disease after ischemia/reperfusion injury" was published in 2022. Journal: Front Nutr.

**FIGURE 9:** Immunohistochemical analysis for α-smooth muscle actin (α-SMA) expression in the renal cortex evaluated after the 90-day protocol in rats submitted to renal ischemia-reperfusion insult on day 45 treated with standard diet (SD), vitamin D-free diet (VDD), high-fat diet (HFD) or high-fat vitamin D-free diet (HFDV). **(A)** Bar graph of α-SMA expression values. **(B)** Representative photomicrographs of immunostaining for α-SMA in the renal cortex from an SD, VDD, HFD, and HFDV rat (400×). Data are mean ± SEM. ^a^*p* < 0.001 and ^c^*p* < 0.05 *vs.* SD; ^d^*p* < 0.001 and ^f^*p* < 0.05 *vs.* VDD; ^i^*p* < 0.05 *vs*. HFD.

**FIGURE 10:** Immunohistochemical analysis for vimentin expression in the renal cortex evaluated after the 90-day protocol in rats submitted to renal ischemia-reperfusion insult on day 45 treated with standard diet (SD), vitamin D-free diet (VDD), high-fat diet (HFD) or high-fat vitamin D-free diet (HFDV). **(A)** Bar graph of vimentin expression values. **(B)** Representative photomicrographs of immunostaining for vimentin in the renal cortex from an SD, VDD, HFD, and HFDV rat (400×). Data are mean ± SEM. ^c^*p* < 0.05 *vs*. SD.

### Adipose tissue and vitamin D roles on the cell proliferation, glomerular vascular endothelium, and tubulointerstitial alterations

The process of epithelial–mesenchymal transition (EMT) promotes greater cell division, allows cells to acquire a secretory phenotype, and contributes to greater deposition of ECM components. After our studies regarding ECM proteins and markers of phenotypical alterations, we proposed to investigate the proliferation of renal cells as well as the integrity of the glomerular vascular endothelium. Initially, we assessed the cell proliferation by evaluating the immunostaining for PCNA in the renal cortex. We verified a higher renal expression of PCNA (%) in the HFDV group (*p* < 0.05) compared to all the other groups (Figure 11). As a marker of glomerular vascular endothelium, we performed IHC studies using an antibody against JG12. Our data revealed a lower JG12 staining (*p* < 0.001) per glomerular tuft area (%) in the VDD and HFD groups compared to the SD group. This alteration was even more evident in the HFDV group, which showed a remarkable reduction in the expression of JG12 in comparison to all the other groups (Figure 12). We found no differences among the groups concerning the glomerular tuft area used to correct the expression of JG12 (Table 2).

**FIGURE 11:** Immunohistochemical analysis for proliferating cell nuclear antigen (PCNA) expression in the renal cortex evaluated after the 90-day protocol in rats submitted to renal ischemia-reperfusion insult on day 45 treated with standard diet (SD), vitamin D-free diet (VDD), high-fat diet (HFD), or high-fat vitamin D-free diet (HFDV). **(A)** Bar graph of PCNA expression values. **(B)** Representative photomicrographs of immunostaining for PCNA in the renal cortex from an SD, VDD, HFD, and HFDV rat (×400). Data are mean ± SEM. ^c^*p* < 0.05 *vs.* SD; ^f^*p* < 0.05 *vs*. VDD; ^i^*p* < 0.05 *vs*. HFD.

The article "The association between obesity and vitamin D deficiency modifies the progression of kidney disease after ischemia/reperfusion injury" was published in 2022. Journal: Front Nutr.

**FIGURE 12:** Immunohistochemical analysis for aminopeptidase P (JG12) expression by glomerular tuft area in the renal tissue evaluated after the 90-day protocol in rats submitted to renal ischemia-reperfusion insult on day 45 treated with standard diet (SD), vitamin D-free diet (VDD), high-fat diet (HFD) or high-fat vitamin D-free diet (HFDV). **(A)** Bar graph of JG12 expression values. **(B)** Representative photomicrographs of immunostaining for JG12 in the renal cortex from an SD, VDD, HFD, and HFDV rat (×400). Data are mean ± SEM. ^a^*p* < 0.001 *vs.* SD; ^f^*p* < 0.05 *vs*. VDD; ^i^*p* < 0.05 *vs*. HFD.

Finally, we evaluated the tubulointerstitial involvement based on our dataset which included the results obtained from the experiments regarding the inflammatory infiltrate, RFF, and consequent interstitial expansion. By histomorphometry, we evaluated the FIA in the renal cortex. The histomorphometric studies revealed an upward tendency regarding FIA in the VDD group in relation to the SD group. In addition, we observed a larger FIA (*p* < 0.05) in the HFD group than in the SD group. Of note, the HFDV group showed a more evident increase (*p* < 0.001) in the FIA compared to all the other groups (Figure 13), which indicates a synergistic role of vitamin D and adipose tissue on the alterations of the tubulointerstitial compartment.

**FIGURE 13:** Fractional interstitial area (FIA) of the renal cortex evaluated after the 90-day protocol in rats submitted to renal ischemia-reperfusion insult on day 45 treated with standard diet (SD), vitamin D-free diet (VDD), high-fat diet (HFD) or high-fat vitamin D-free diet (HFDV). **(A)** Bar graph of FIA values. **(B)** Masson’s trichrome representative photomicrographs of renal histological changes from an SD, VDD, HFD, and HFDV rat (×400). Data are mean ± SEM. ^a^*p* < 0.001 and ^c^*p* < 0.05 *vs.* SD; ^d^*p* < 0.001 *vs.* VDD; ^g^*p* < 0.001 *vs.* HFD.

## Discussion

Our results show that the animals fed a high-fat vitamin D-free diet and submitted to renal IRI presented almost undetectable levels of vitamin D and changes in the anthropometric and metabolic profile. The combination of vitamin D deficiency and obesity modified functional and hemodynamic parameters. Furthermore, we observed an increase in proteinuria, renal expression of MCP-1, infiltration of inflammatory cells, ECM proteins, and phenotypical markers in the HFDV. This group also presented a greater cell proliferation, impairment of the glomerular vascular endothelium, and expansion of the tubulointerstitial compartment. All those alterations were associated with a higher expression of TGF-β1 and a lower expression of VDR in the renal tissue from the HFDV group.

The article "The association between obesity and vitamin D deficiency modifies the progression of kidney disease after ischemia/reperfusion injury" was published in 2022. Journal: Front Nutr.

Plasma levels of vitamin D represent the sum of biological production from diet and sun exposure (38). It is important to state that our animals were kept without sun exposure and received diets depleted or not in vitamin D. The vitamin D-free diet groups (VDD and HFDV) had almost undetectable plasma levels of vitamin D at the end of the 90-day protocol, confirming the efficiency of the experimental model of vitamin D deficiency (2, 6, 8). Plasma levels of vitamin D have been inversely associated with obesity, insulin resistance, and type 2 diabetes (12, 15, 39). In addition to the HFDV rats, we observed lower plasma levels of vitamin D as well as a downward tendency regarding the renal expression of VDR in the HFD rats. Our results are consistent with the hypothesis of a lower and inadequate bioavailability of vitamin D in obesity (12, 15, 39).

Usually considered a storage organ for vitamin D, adipose tissue also seems to influence endocrine and paracrine actions, modulating the expression of enzymes responsible for the formation, activation, and degradation of vitamin D (12, 40, 41). Besides the renal protein expression, we evaluated VDR gene expression in the adipose tissue. Our VDD group showed a lower VDR gene expression, which primarily followed the deficient plasma levels of vitamin D. In 2015, Nguyen et al. described the association between plasma vitamin D levels and VDR gene expression in adipose tissue (39). However, we did not observe this relationship in our HFDV rats. Even receiving a vitamin D-depleted diet, HFDV rats showed a higher renal expression of VDR and a marked gene expression of this receptor in adipose tissue compared to VDD rats. In addition, our groups that received the high-fat diets (HFD and HFDV) showed a downward tendency in the VDR gene expression in adipose tissue in relation to the SD group. Wamberg et al. also observed a reduced VDR gene expression in the subcutaneous adipose tissue of obese women in comparison to lean individuals. On the other hand, these authors demonstrated that there was a 33% higher expression of VDR in the visceral adipose tissue of obese women compared to lean women (41). Nevertheless, our results are not enough to understand the physiological actions of vitamin D on adipose tissue associated with the degree of obesity and future studies are needed to explain this relationship.

The article "The association between obesity and vitamin D deficiency modifies the progression of kidney disease after ischemia/reperfusion injury" was published in 2022. Journal: Front Nutr.

Hypercaloric and high-fat diets are described in the literature as being effective for the experimental induction of obesity in rodents (42–44). As a confirmation of the effectiveness of our experimental model, the anthropometric measurements used as markers of obesity demonstrated that HFD and HFDV rats presented higher body weight and BMI as well as a significant increase in their abdominal and thoracic circumferences.

Hyperlipidemia is commonly related to a high intake of diets rich in fatty acids and obesity (45, 46). It is described that the abnormal deposition of fat in adipose tissue and in other organs, such as the liver and kidneys, can be considered an important risk in the follow-up of pathologies, including CKD (45, 47, 48). The presence of dyslipidemia is reported in all stages of CKD, with impairment of the glomerular filtration barrier, tubular damage, and proteinuria (47). Our HFD and HFDV rats showed higher plasma levels of cholesterol and triglycerides than SD and VDD rats. Bhandari et al. also showed the adverse effects of obesity induced by a high-fat diet. Corroborating our data, these authors demonstrated alterations in the lipid profile of rodents, such as the presence of high levels of total cholesterol, triglycerides, and LDL, followed by low levels of HDL (43).

The relationship between lipid profile and vitamin D is also demonstrated in the literature (6, 49, 50). It has been reported that vitamin D and cholesterol share the same biosynthesis pathway, as they have 7-dehydroxycholesterol as a common precursor (46). In the present study, the vitamin D-deficient rats, particularly HFDV rats, had higher levels of cholesterol associated with remarkable triglyceride levels compared to SD animals. Vitamin D plays important roles in the regulation and absorption of calcium, thus reducing the absorption of fatty acids and exerting an influence on plasma cholesterol levels (51). In addition, low levels of vitamin D promote plasma PTH elevation. High levels of PTH increase lipogenesis, and bone remodeling, and reduce lipolytic activity, thus influencing lipid metabolism (46, 48, 51). As expected, our VDD and HFDV groups presented elevated PTH levels in relation to SD and HFD groups, demonstrating the negative feedback caused by vitamin D deficiency.

Hyperglycemia is a typical sign of both reduced gluconeogenesis in the liver and reduced glucose uptake in skeletal muscle, liver, and adipose tissue, which feature the onset of insulin resistance (50, 52). In addition to overweight, increased visceral adipose tissue represents an important association with insulin resistance and changes in adipose tissue functionality (53). Vitamin D deficiency is also related to inadequate insulin secretion, altered blood glucose levels, and type 2 diabetes (54–57). One of the mechanisms by which hypovitaminosis D contributes to the installation of insulin resistance is *via* the regulation of intracellular calcium in pancreatic β-cells (50, 58). In the present study, we found an upward tendency in fasting plasma glucose in VDD and HDF groups. Simultaneously, the association between obesity and vitamin D deficiency promoted a higher glycemia in the HFDV group in comparison to all the other groups. Thereby our dataset regarding the metabolic parameters (cholesterol, triglycerides, and fasting blood glucose) allowed us to observe the influence of obesity and vitamin D deficiency, alone or in association, on the installation of metabolic syndrome, especially in the HFDV animals.

The article "The association between obesity and vitamin D deficiency modifies the progression of kidney disease after ischemia/reperfusion injury" was published in 2022. Journal: Front Nutr.

Adipose tissue is not only recognized for its capacity for energy storage and lipid mobilization, but also as an adipokine-secreting endocrine organ (22, 53). It is known that adipocytes, one of the main cell types of the adipose tissue, secrete a variety of factors and hormones, such as TNF-α, IL-6, PAI-1, MCP-1, adiponectin, resistin, and leptin (22, 23, 59). Physiologically, leptin plays an important role in the control of energy homeostasis and maintenance of body weight, with circulating levels proportional to food intake and body energy reserve from the suppression or activation of specific neurotransmitters (60, 61). The condition called hyperleptinemia in obesity induces leptin resistance, which is similar to insulin resistance in type 2 diabetes (61). In the present study, our HFD and HFDV groups showed higher plasma leptin levels than the SD group. Corroborating our results, previous studies also showed an increase in serum leptin levels in experimental models of obesity induced by high-fat diets (62–64). In addition to being directly related to the amount of adipose tissue, leptin concentration seems to be also regulated by serum vitamin D levels (65, 66). Conversely, leptin appears to have an inhibitory effect on the conversion of 25(OH)D to 1,25(OH)_2_D_3_, by inhibiting 1-α-hydroxylase in renal and adipose tissue (66, 67). Those findings are in agreement with our data regarding the notorious high plasma leptin levels observed in the HFDV rats. Thus, our results allow us to infer that the synergistic effect of vitamin D deficiency and obesity could explain the significant increase in plasma leptin levels observed in the HFDV group.

It is well known that CKD, even in the early stages, is accompanied by a progressive decline in GFR and low levels of vitamin D (1, 7, 8, 10, 68). In 2011, de Boer et al. suggested that vitamin D deficiency may be a risk factor for the decline in GFR, especially when associated with diabetes and hypertension (69). Our VDD rats presented a lower GFR compared to SD and HFD rats, confirming previous results from our group regarding the role of vitamin D deficiency on the impairment of the renal function (1, 7, 8). In addition, obesity and dyslipidemia are described as aggravating factors in the progression of kidney disease, promoting damage to the glomerular filtration barrier and the subsequent presence of proteinuria (25, 47, 70, 71). Although not significant, the HFDV group presented a decrease of ∼13% in GFR in relation to VDD group and a greater proteinuria than the HFD group. Associated with these results, the HFDV group also presented a lower glomerular expression of JG12 compared to all the other groups. Corroborating these results, previous studies from our laboratory demonstrated a decreased renal JG12 expression in vitamin D-deficient rats in renal IRI and 5/6 nephrectomy model (7, 8). Since JG12 is an aminopeptidase responsible for anchoring the cells in the cell membrane, it is plausible to infer that the lower expression of this protein might have contributed to the impaired renal function observed in the HFDV group. Taken together, those results suggest that either isolated or combined effects of obesity and vitamin D deficiency may impair renal function.

The article "The association between obesity and vitamin D deficiency modifies the progression of kidney disease after ischemia/reperfusion injury" was published in 2022. Journal: Front Nutr.

It is common knowledge that the RAAS is responsible for maintaining vascular resistance and extracellular fluid homeostasis (72). The negative endocrine regulation of the RAAS by vitamin D is demonstrated in the literature mainly by an inverse relation of this hormone levels and the expression of renin (72, 73). This impairment of systemic blood pressure control generated by hypovitaminosis D has also been demonstrated in previous studies from our group, which associated changes in the activation of the RAAS with alterations in endothelium and renal vasculature (1, 2, 7, 72–74). Furthermore, the association between obesity and increased MAP has been suggested as an important link in kidney injury (5). In the present study, we found a higher MAP as well as increased plasma levels of Ang II and aldosterone in the VDD, HFD, and HFDV groups, suggesting a greater activation of the RAAS. The main mechanisms involved in the elevation of MAP levels in the course of obesity are described as: (1) activation of the sympathetic nervous system by increasing intra-abdominal pressure and higher levels of leptin; (2) RAAS activation due to increased secretion of inflammatory cytokines such as TNF-α, IL-6, resistin, and leptin by adipocytes; (3) increased aldosterone levels by leptin stimulation to the adrenal gland, increasing Na+ retention and plasma volume expansion; and (4) reduced adiponectin expression, which appears to be one of the causes of increased inflammation in obesity (5, 26, 75, 76). Our data showed that the association between obesity and vitamin D deficiency potentiated hemodynamic impairment. Collectively, changes in MAP and plasma levels of Ang II/aldosterone as well as in RBF and RVR support the hemodynamic disturbance observed in the HFDV group.

The article "The association between obesity and vitamin D deficiency modifies the progression of kidney disease after ischemia/reperfusion injury" was published in 2022. Journal: Front Nutr.

Inflammatory cells including macrophages and T cells play a key role in tissue homeostasis and immune responses, especially in the course of kidney diseases (7, 77). Moreover, an exacerbated inflammatory response is usually associated with a growing RFF (7, 77). This process involves several steps, including the stimulation of cell division and the production of chemokines to recruit cells to the site of injury (78). In addition to a higher renal expression of MCP-1 and CD68+ cells, our HFD group presented an upward tendency regarding the expression of CD3+ cells in relation to the SD group, which demonstrates a possible influence of adipose tissue on the inflammatory response. Corroborating our results, Decleves et al. also observed increased renal and urinary expression of MCP-1 in mice fed a high-fat diet (35). In the present study, we also observed similar results concerning the renal expression of MCP-1, CD3+, and CD68+ cells in the VDD group, reinforcing the immunomodulatory effect of vitamin D (1, 7, 77). Of note, we found a higher renal expression of MCP-1, CD3+, and CD68+ cells in the HFDV group compared to all the other groups, demonstrating a synergistic effect of adipose tissue and vitamin D deficiency regarding the inflammatory process.

Macrophage activation and function are heterogeneous and regulated by the microenvironment and stage of tissue injury, reflecting in different phenotypes (1, 77, 79). In general, macrophages are classified into two subtypes: (a) M1 macrophages, classically activated and considered pro-inflammatory due to their ability to produce and release pro-inflammatory cytokines, such as IL-1, IL-6, IL-12, IL- 23, and TNF-α; and (b) M2 macrophages, which are known to have anti-inflammatory and immunomodulatory functions (79, 80). In the present study, we observed a higher renal expression of CD68+ cells (M1+M2 macrophages) in the VDD, HFD, and HFDV groups compared to the SD group. In addition, we noted an upward tendency concerning the expression of those cells in the HFDV group. Although not significant, we noticed a lower renal expression of CD206+ cells (M2 macrophages) in relation to the total amount of CD68+ cells in the HFDV group. It is reported that the balance between M1/M2 macrophages is related to the renal microenvironment and may influence the progression of renal disease (1, 77, 80). In previous studies, we demonstrated that vitamin D deficiency contributed to the extension of the active state of inflammation, reinforcing the role of vitamin D in the modulation of inflammatory cells (1, 7, 77). Concurrently, macrophage infiltration is correlated with the degree of obesity, mainly with the M1 phenotype (79). The inflammatory cytokines produced by M1 macrophages neutralize the insulin-sensitizing actions of the hormones adiponectin and leptin, which eventually lead to insulin resistance (79). In contrast, macrophages in lean subjects express high levels of M2-specific genes, such as IL-10 and Arg-1 (79). Thus, our results show that the association between obesity and vitamin D deficiency contributed to an exacerbation of the inflammatory process observed in the HFDV group, which had higher expression of MCP-1 and CD3+ cells and a lower proportion of CD206+ cells in relation to the CD68+ cells.

The article "The association between obesity and vitamin D deficiency modifies the progression of kidney disease after ischemia/reperfusion injury" was published in 2022. Journal: Front Nutr.

As previously reported, AKI can result in incomplete tissue repair, persistent tubulointerstitial inflammation, fibroblast proliferation, and excessive deposition of ECM components (81). Furthermore, in response to kidney injury, cells that are normally stably differentiated to promote homeostasis can dedifferentiate into a new phenotype and redirect tissue repair in a process known as EMT (78). High-fat diets seem to be associated with susceptibility to RFF through increased expression of TGF-β and ECM components (36, 82). Furthermore, studies have shown that vitamin D can suppress the expression of TGF-β and its respective receptor and inhibit the EMT process, cell proliferation, and apoptosis as well (1, 2, 37). Corroborating those findings, we observed a higher renal expression of TGF-β1 in the VDD and HFD groups compared to the SD group. Importantly, the HFDV group presented a higher expression of TGF-β1 than all the other groups, which was associated with higher amounts of Col-3 and fibronectin in the renal tissue. These results suggest the interaction between obesity and vitamin D deficiency on the renal TGF-β1 expression and ECM production.

As aforementioned, EMT process promotes greater cell division, allows cells to acquire a secretory phenotype, and contributes to greater deposition of ECM components (78, 83). In 2012, Xiong et al. reported that the low expression of VDR in CKD would be involved in the relationship between inflammation and EMT (84). In the present study, we observed a higher renal expression of PCNA, α-SMA, and vimentin in the renal cortex from the HFDV group. Previous studies from our laboratory demonstrated the influence of vitamin D deficiency on increased phenotypic change (2) and cell proliferation (8). Corroborating our results regarding obesity, Coimbra et al. also observed a higher expression of vimentin in the renal tissue of obese Zucker rats (85). Furthermore, Amaral et al. showed a higher PCNA expression in the renal cortex of ovariectomized rats in obesity induced by a high-fat diet (86). Thus, similar to our data regarding ECM markers, our results suggest that the synergistic effect of obesity and vitamin D deficiency exacerbated cell proliferation and phenotype alteration of renal tubule cells in the HFDV group.

The article "The association between obesity and vitamin D deficiency modifies the progression of kidney disease after ischemia/reperfusion injury" was published in 2022. Journal: Front Nutr.

Fibrosis and inflammation are hallmarks in the course of kidney disease, in which unresolved kidney inflammation becomes an important driving force for the RFF (1, 87, 88). Some studies have been demonstrating that sufficient levels of vitamin D exert a protective effect in preserving cell integrity. Moreover, those reports show that a close relationship among vitamin D levels, VDR expression, and TGF-β could be involved in inflammation and EMT process (2, 37, 84). Previous data from our group showed that vitamin D deficiency caused a lower renal VDR expression and a higher renal TGF-β1 expression in rats submitted to renal IRI (2) and 5/6 nephrectomy (7, 77). Concomitantly, adipose tissue is recognized as an endocrine organ involved in the production and action of adipokines, including leptin, TNF-α, MCP-1, and TGF-β (23, 70, 89). In the present study, along with the increased expression of TGF-β1 and leptin as well as the decreased expression of the VDR, the HFDV group presented an exacerbated inflammatory infiltrate, greater cell proliferation, and phenotypic alteration of renal tubular cells. Taken together, these changes reflected a significant enlargement of the FIA in the HFDV group. Those results demonstrated a plausible synergistic effect of increased production and secretion of adipokines by adipose tissue and an impaired renoprotective action attributed to hypovitaminosis D. Hence, our data demonstrated that obesity associated with vitamin D deficiency led to a potentiation of the expression of inflammatory and pro-fibrotic factors in the progression following AKI induced by renal IRI.

Our results allow us to conclude that the association between vitamin D deficiency and obesity in the renal ischemia/reperfusion model modified functional, hemodynamic, and metabolic parameters and contributed to a greater expression of inflammatory and pro-fibrotic factors related to the progression of renal disease.

The article "The association between obesity and vitamin D deficiency modifies the progression of kidney disease after ischemia/reperfusion injury" was published in 2022. Journal: Front Nutr.

## Data availability statement

The original contributions presented in this study are included in the article/supplementary material, further inquiries can be directed to the corresponding author.

## Ethics statement

The animal study was reviewed and approved by Research Ethics Committee of Faculty of Medicine, University of São Paulo (CEUA, registration 1438/2020).

## Author contributions

DB, DC, MN, MS, AB, and RV: performed the experiments. DB, DC, AB, and RV: analyzed the data and contributed to the writing of the manuscript. All authors conceived and designed the experiments, reviewed the manuscript, and approved the submitted version.
